The article "Protective Effects of Soy Oligopeptides in Ultraviolet B-Induced Acute Photodamage of Human Skin" was retracted in 2020. Reason: duplicated images.

# Protective Effects of Soy Oligopeptides in Ultraviolet B-Induced Acute Photodamage of Human Skin

**DOI:** 10.1155/2016/5846865

**Published:** 2016-07-12

**Authors:** Bing-rong Zhou, Li-wen Ma, Juan Liu, Jia-an Zhang, Yang Xu, Di Wu, Felicia Permatasari, Dan Luo

**Affiliations:** Department of Dermatology, The First Affiliated Hospital of Nanjing Medical University, Nanjing 210029, China

## Abstract

*Aim*. We explored the effects of soy oligopeptides (SOP) in ultraviolet B- (UVB-) induced acute photodamage of human skin* in vivo* and foreskin* ex vivo*.* Methods*. We irradiated the forearm with 1.5 minimal erythemal dose (MED) of UVB for 3 consecutive days, establishing acute photodamage of skin, and topically applied SOP. Erythema index (EI), melanin index, stratum corneum hydration, and transepidermal water loss were measured by using Multiprobe Adapter 9 device. We irradiated foreskin* ex vivo* with the same dose of UVB (180 mJ/cm^2^) for 3 consecutive days and topically applied SOP. Sunburn cells were detected by using hematoxylin and eosin staining. Apoptotic cells were detected by using terminal deoxynucleotidyl transferase dUTP nick end labeling assay. Cyclobutane pyrimidine dimers (CPDs), p53 protein, Bax protein, and Bcl-2 protein were detected by using immunohistochemical staining.* Results*. Compared with UVB group, UVB-irradiated skin with topically applied SOP showed significantly decreased EI. Compared with UVB group, topical SOP significantly increased Bcl-2 protein expression and decreased CPDs-positive cells, sunburn cells, apoptotic cells, p53 protein expression, and Bax protein expressions in the epidermis of UVB-irradiated foreskin.* Conclusion*. Our study demonstrated that topical SOP can protect human skin against UVB-induced photodamage.

## 1. Introduction

When the skin receives more than the maximum tolerated dose of ultraviolet (UV) irradiation, an acute phototoxic reaction can occur. Ultraviolet B (UVB) can induce 100–800 times greater biological effects in the skin compared with ultraviolet A (UVA) of the same dose, and the most visual indicator of acute injury to skin caused by UVB is erythema. During erythema formation, there is infiltration of inflammatory cells in the dermis and sunburn cells in the epidermis. Sunburn cells are apoptotic keratinocytes, which show nuclear shrinkage and uniform cytoplasm and are eosinophilic and deeply stained. Sunburn cell formation is a defense mechanism for preventing malignant changes of epithelial cells [1].

Pyrimidine (6-4) pyrimidone photoproducts (6-4PPs) and cyclobutane pyrimidine dimers (CPDs) are two major types of DNA lesions induced by UVB [2]. CPDs are formed more abundantly and repaired less efficiently than the 6-4PPs and are therefore considered as the predominant UVB-induced DNA photolesions [2, 3]. If DNA lesions cannot be repaired in time, UVB-damaged cells will be removed by apoptosis, and p53 tumor suppressor protein is the key regulatory factor of apoptosis [4–6].

The article "Protective Effects of Soy Oligopeptides in Ultraviolet B-Induced Acute Photodamage of Human Skin" was retracted in 2020. Reason: duplicated images.

Soy oligopeptides (SOP) are hydrolysates obtained from proteolytic hydrolysis of soybean proteins, consisting of 3–6 amino acids with <1000 low molecular weight peptides, mainly 300–700 kDa [7]. Recently, various biological functions of soybean oligopeptides have been found such as antioxidant, blood pressure lowering, and blood lipid lowering effects [8, 9]. Our previous study (written in Chinese) has confirmed that soybean oligopeptides could effectively relieve photodamage induced by UVB irradiation in mice [10].

In this study, we conducted* in vivo* and* ex vivo* studies using human skin. In a clinical study, we topically applied SOP on UVB-irradiated forearm skin. We evaluated the erythema index (EI), melanin index (MI), transepidermal water loss (TEWL), and stratum corneum (SC) hydration of the irradiated skin at certain time points. In an* ex vivo* study, we applied SOP on UVB-irradiated foreskin. We detected sunburn cells, apoptotic cells, p53 protein, Bax protein, Bcl-2 protein, and CPDs. We aimed to evaluate the effects of SOP in UVB-irradiated human skin and the underlying mechanisms.

## 2. Materials and Methods

### 2.1. Ethics Statement

This study was approved by the institutional review board of Nanjing Medical University, Nanjing, China (approval number 2013-SRFA-025). Written informed consent was obtained from all participants before taking part in this research.

### 2.2. SOP Preparation

SOP was prepared from soybean protein isolates (SPI) obtained from Jilin Fuji Protein Co. Ltd. (Jilin, China), as described previously [11]. Alcalase (obtained from Novozymes Biological Co., Tianjin, China) at a ratio of 600,000 U/kg (enzyme/protein substrate) was added to the solution and the hydrolysis was kept at pH 8.5 by continuous addition of 20% NaOH. The degree of hydrolysis (DH) of soybean protein was calculated by using the pH stat method. After the DH reached around 10–15%, the suspension was cooled down to 50°C and added with Protex 13 FL (purchased from Genencor, Division of Danisco, Wuxi, China) at a ratio of 200,000 U/kg (enzyme/protein substrate). Then, the mixture was incubated at 50°C until the DH reached 20–25%. The reaction was stopped by heating the mixture to 90°C for 15 min to inactivate the enzyme, and the resulting hydrolysate was centrifuged at 15,000 ×g for 10 min (SYGQ105 tube centrifuge, Shanghai Shiyuan Bioengineering Equipment Co., Shanghai, China). The supernatant was filtered with UF-5000 ultrafiltration equipment (molecular weight cut-off 5,000 Da, Xinda Membrane Tech. Co., Hefei, China) and then evaporated with a double-effect falling film evaporator (OE2, OECH Machinery Equipment Co., Ltd., Hefei, China) at 0.10 ± 0.02 MPa and 60 ± 5°C, until the solid content of the concentrated liquid reached 30–40%. The concentrated solution containing peptides was dried with a spray drier (YG30, Wuxi City Sunlight Drier Factory, Wuxi, China) at a 15 kg/h flow rate with inlet temperature of 160–180°C and outlet temperature of 80–90°C. The peptides present in SOP extract were analyzed and quantified using HPLC. The peptide and free amino acid contents of SOP were 82.5 ± 1.13% and 3.7 ± 0.28%, respectively. The molecular weight distribution of SOP was mainly below 1,000 Da (85.4%), 56.7% of which were 140–500 Da. SOP creams were custom-order produced by Infinitus Ltd., China, and were used for* in vivo* and* ex vivo* experiments.

The article "Protective Effects of Soy Oligopeptides in Ultraviolet B-Induced Acute Photodamage of Human Skin" was retracted in 2020. Reason: duplicated images.

### 2.3. *In Vivo* Study Protocol

#### 2.3.1. Volunteer Recruitment

Nine healthy male volunteers who were in the range from 23 to 26 years old with Fitzpatrick skin types III to IV were enrolled in the study. All volunteers had no light-related skin and systemic diseases. All volunteers denied any drug use in the past month prior to and throughout the experiment. Sunlight exposure on the experimental site was avoided throughout the experiment.

#### 2.3.2. Group Division and Treatments

The flexor side of the left forearm was selected as the experimental site. The selected UVB dose was 180 mJ/cm^2^. There were eight areas of 1.5 cm × 1.5 cm designated as the following 8 groups: (1) negative control group; (2) vehicle control group; (3) SOP group; (4) UVB group; (5) UVB + vehicle group; (6) UVB + 2.5 IU/mL SOP group; (7) UVB + 5.0 IU/mL SOP group; (8) UVB + 10.0 IU/mL SOP group. Hence, UVB dose = UVB irradiation intensity × irradiation time (s). The UVB irradiation apparatus was from Sigma High-Tech Co., Ltd. (Shanghai, China). UVB irradiation was delivered by using a Philips TL 20W/12 (Eindhoven, Netherlands) at an intensity of 1.5 mW/cm^2^, a fluorescent bulb emitting 280–320 nm wavelength with a peak at 313 nm. Irradiation output was monitored using a UV-meter (Waldmann, Villingen-Schwenningen, Germany).

Five minutes after irradiation with 180 mJ/cm^2^ UVB, SOP cream (provided by Infinitus Ltd., China) at 3 different concentrations (2.5, 5.0, and 10.0 IU/mL) was topically applied on the selected areas. This procedure was done for 3 consecutive days. MI, EI, TEWL, and SC hydration were detected 1, 3, and 10 days after the last treatment.

The article "Protective Effects of Soy Oligopeptides in Ultraviolet B-Induced Acute Photodamage of Human Skin" was retracted in 2020. Reason: duplicated images.

#### 2.3.3. Detection of Skin Indexes Using Multifunctional Skin Test

The experimental site was cleansed with warm water, free from skin care products or drugs, and the volunteers were requested to have a seat and rest for 2 hours. The experimental site was then examined using Multiprobe Adapter (MPA) 9 device (CK Electronic, Germany) in a room with no direct sunlight and ventilation at a room temperature of 25-26°C and relative humidity of 50–60%. MI and EI were detected using Mexameter MX 18 probe, TEWL was detected using Tewameter TM 300 probe, and SC hydration was detected using Corneometer CM 825 probe. The instrument used in the present study has been sent to the manufacturer for calibration biannually.

### 2.4. *Ex Vivo* Study Protocol

#### 2.4.1. Foreskin Preparation

Fresh and healthy foreskins from 20 cases (ages ranged from 20 to 30 years) were obtained by circumcisions as approved by the Ethics Committee in the First Affiliated Hospital of Nanjing Medical University (Nanjing, China). The subcutaneous tissue was removed by scraping with forceps. The foreskin was washed 3 times with saline, each time for 3 minutes. The foreskin was cut into 4 parts and the size of each part was 0.5 cm × 1.0 cm. Roswell Park Memorial Institute (RPMI) medium (containing 10% fetal bovine serum (FBS), 2 mM glutamine, 100 U/mL penicillin, 100 *μ*g/mL streptomycin, and 20 *μ*M *β*-mercaptoethanol) was added to a Petri dish. The foreskin was placed into the Petri dish with the dermis facing downwards and the bottom immersed in the culture medium, whilst the epidermis was above the culture medium surface [12].

#### 2.4.2. Group Division

The foreskins were randomly divided into 4 groups: (1) control group; (2) UVB group; (3) UVB + vehicle group; (4) UVB + 5.0 IU/mL SOP group. Each group was detected at 4 different time points (8, 24, 48, and 72 h after UVB irradiation).

#### 2.4.3. UVB Irradiation and SOP Application* Ex Vivo*

UVB groups, UVB + vehicle groups, and UVB + SOP groups were placed into 24-well culture dish. The epidermal side of the foreskin was irradiated once by UVB at a dose of 180 mJ/cm^2^ and an intensity of 1.5 mW/cm^2^. 5 min after UVB irradiation, SOP cream was applied evenly on the epidermis of the foreskin by using a sterile cotton swab. Each foreskin was divided into 4 parts, immersed in the culture medium, and placed in the 37°C incubator for different times (8, 24, 48, or 72 h).

#### 2.4.4. Histopathology Using Hematoxylin and Eosin (H&E) Staining

Tissues were fixed in 10% formalin and embedded in paraffin. Vertical sections (6 *μ*m) were cut, mounted on glass slides, and stained with H&E. Microscopic evaluation (Olympus, Japan) and digital photography of the slides were taken. The mean number of sunburn cells (with a pyknotic nucleus and densely stained eosinophilic cytoplasm) was quantified in five random fields at 400 times magnification.

The article "Protective Effects of Soy Oligopeptides in Ultraviolet B-Induced Acute Photodamage of Human Skin" was retracted in 2020. Reason: duplicated images.

#### 2.4.5. TUNEL Assay

To evaluate apoptosis, Terminal dUTP Nicked Labelling was used as a marker for apoptosis. TUNEL* in situ* detection kit was purchased from KeyGen Biotech, China. In brief, tissue sections (5 *μ*m) after deparaffinization and re-hydration were permeabilized with proteinase K (30 mg/mL) for 1 h at 37°C. Thereafter, the sections were quenched of endogenous peroxidase activity using 3% hydrogen peroxide for 10 min. After thorough washing with 1x PBS, sections were incubated with equilibration buffer for 10 min, and then the TdT reaction mixture was added to the sections, except for the negative control, and incubated at 37°C for 1 h. The reaction was stopped by immersing the sections in 2x saline– sodium citrate buffer for 15 min. Sections were then added with streptavidin– HRP (1 : 500) for 30 min at room temperature, and after repeated washings, sections were incubated with substrate DAB until color development. The micrographs were obtained using a light microscope (Olympus, Japan) and the mean level of apoptotic cells (with brown granules in the nucleus) was quantified in five random fields at ×400 magnification.

#### 2.4.6. Immunohistochemical Staining

Briefly, skin samples were processed conventionally before paraffin embedding, and serial 4 *μ*m sections were cut and were deparaffinized and rehydrated with water. Endogenous peroxidase activity was blocked by 10 min incubation with 3% hydrogen peroxide, and slides were then incubated with 0.125% trypsin for 10 min at 37°C and then with 1 N HCl for 30 min at room temperature. Slides were washed with PBS and then incubated for 30 min with 10% goat serum in PBS. Sections were then incubated with CPDs-specific monoclonal antibody (Sigma Co. Ltd., St. Louis, MO, USA), p53-specific monoclonal antibody (Sigma Co. Ltd., St. Louis, MO, USA), Bax-specific monoclonal antibody (Santa Cruz Co., USA), and Bcl-2-specific monoclonal antibody (Santa Cruz Co., USA). Bound anti-CPDs antibody was detected by incubation with biotinylated goat anti-mouse IgG1 followed by peroxidase-labeled streptavidin. Slides were developed with 3,30-diaminobenzidine (DAB, Fuzhou Maixin Biotech. Co., Ltd.) as a substrate for 3–5 min. The sections were then rinsed with distilled water and counterstained with H&E, cleared, and mounted. The DAB-peroxidase reaction gave a brown reaction product. The mean level of CPDs and p53-positive cells was quantified under a light microscope (Olympus, Japan) in five random fields at ×400 magnification. Bax was mainly expressed as brownish materials in the cytoplasm. Bcl-2 was localized in the cytoplasm and cell membrane.

The article "Protective Effects of Soy Oligopeptides in Ultraviolet B-Induced Acute Photodamage of Human Skin" was retracted in 2020. Reason: duplicated images.

#### 2.4.7. Immunohistochemical Analysis

Immunohistochemical evaluation was done as described by Bayramgürler et al. [13]. The proportion of the immunoreactive cells was assessed as follows: 0 meant there are no immunoreactive cells; 1 meant 1–25% of the cells are immunoreactive; 2 meant 26–50% of the cells are immunoreactive; 3 meant 51–75% of the cells are immunoreactive; 4 meant more than 75% of the cells are immunoreactive. The staining intensity of the cells was graded as 0 (no staining), 1 (light staining), 2 (moderate staining), and 3 (intense staining). An immunoreactivity intensity distribution index (IRIDI) was calculated as follows: the score of the staining intensity multiplied by the score of the proportion of the immunoreactive cells.

### 2.5. Statistical Analysis

Statistical analysis was performed by using SPSS for Windows version 16.0 (SPSS, Chicago, IL, USA). The statistical analysis for the* in vivo* study was carried out with the paired *t*-test. The statistical analysis for the* ex vivo* study was carried out with the Kruskal-Wallis *H* test and Mann-Whitney *U* test, and all were two-sided tests. Data were expressed as the mean ± SD for each group. A *P* value of less than 0.05 (*P* < 0.05) was considered statistically significant.

## 3. Results

### 3.1. *In Vivo* Study

#### 3.1.1. The Effect of Topical SOP on the EI of UVB-Irradiated Human Skin

One, three, and ten days after UVB irradiation, the skin EI of all UVB-irradiated groups was significantly increased (*P* < 0.05) compared with negative control group. Compared with UVB group, the skin EI in UVB + 5.0 IU/mL SOP and UVB + 10.0 IU/mL SOP groups was significantly decreased (*P* < 0.05), whilst that of UVB + 2.5 IU/mL SOP group showed no significant difference (*P* > 0.05). The lowest skin EI was achieved by UVB + 5.0 IU/mL SOP group (*P* < 0.05). There was no significant difference in the skin EI among nonirradiated groups (*P* > 0.05) (Figure 1(a)).

#### 3.1.2. The Effect of Topical SOP on the MI of UVB-Irradiated Human Skin

One day after UVB irradiation, there was no significant difference in the skin MI of UVB-irradiated groups compared with negative control group (*P* > 0.05), but it was significantly increased on days 3 and 10 (*P* < 0.05 and *P* < 0.001, resp.). Compared with UVB group, UVB + SOP groups showed no significant difference in the skin MI (*P* > 0.05). There was no significant difference in the skin MI among nonirradiated groups (*P* > 0.05) (Figure 1(b)).

#### 3.1.3. The Effect of Topical SOP on the SC Hydration of UVB-Irradiated Human Skin

One and three days after UVB irradiation, the SC hydration in each irradiated group was significantly decreased (*P* < 0.05) compared with negative control group, but there was no significant difference on day 10 (*P* > 0.05). Compared to UVB group, the SC hydration on day 1 in UVB + 5.0 IU/mL SOP and UVB + 10.0 IU/mL SOP groups was significantly increased (*P* < 0.05), whilst that of days 3 and 10 showed no significant difference (*P* > 0.05). There was no significant difference in the SC hydration among nonirradiated groups (*P* > 0.05) (Figure 1(c)).

The article "Protective Effects of Soy Oligopeptides in Ultraviolet B-Induced Acute Photodamage of Human Skin" was retracted in 2020. Reason: duplicated images.

#### 3.1.4. The Effect of Topical SOP on TEWL of UVB-Irradiated Human Skin

One, three, and ten days after UVB irradiation, the skin TEWL in all UVB-irradiated groups showed no significant difference (*P* > 0.05) compared with negative control group. Compared with UVB group, the skin TEWL in UVB + SOP groups on days 1, 3, and 10 also showed no significant difference (*P* > 0.05). There was no significant difference in the skin TEWL among nonirradiated groups (*P* > 0.05) (Figure 1(d)).

### 3.2. *Ex Vivo* Study

#### 3.2.1. The Effect of Topical SOP on the Proportion of CPDs-Positive Cells in the Epidermis after UVB Irradiation

After UVB irradiation, the epidermis CPDs-positive cells were stained brownish by immunohistochemical staining. There were no CPDs-positive cells in the epidermis of the control group. UVB-irradiated groups showed a large number of CPDs-positive cells in the epidermis, and the highest number was observed at 8 h. Then, 8, 24, 48, and 72 h after UVB irradiation, the proportion of CPDs-positive cells in UVB + SOP groups was significantly decreased compared with UVB group (*P* < 0.05). The difference in the proportion of CPDs-positive cells between UVB + vehicle and UVB groups was not significant (*P* > 0.05) (Figures 2(a) and 2(b)).

#### 3.2.2. The Effect of Topical SOP on the Proportion of Sunburn Cells in the Epidermis after UVB Irradiation

Here, 8, 24, 48, and 72 h after UVB irradiation, there were a large number of sunburn cells in the epidermis of UVB-irradiated groups, and the highest number was observed at 24 h. The proportion of sunburn cells in the epidermis of UVB + SOP groups at 8, 24, 48, and 72 h after UVB irradiation was significantly decreased compared with UVB group (*P* < 0.05). The difference between UVB group and UVB + vehicle groups at different time points was not significant (*P* > 0.05) (Figures 3(a) and 3(b)).

#### 3.2.3. The Effect of Topical SOP on the Proportion of Apoptotic Cells in the Epidermis after UVB Irradiation

The apoptotic cells were stained brown by TUNEL staining. There was no apoptotic cell in the epidermis of the control group. There were a large number of apoptotic cells in the epidermis of UVB-irradiated groups, and the highest number was at 24 h. Compared with UVB group, the proportion of apoptotic cells in UVB + SOP groups at 8, 24, 48, and 72 h was significantly decreased (*P* < 0.05). There was no significant difference between UVB + vehicle and UVB groups (*P* > 0.05) (Figures 4(a) and 4(b)).

The article "Protective Effects of Soy Oligopeptides in Ultraviolet B-Induced Acute Photodamage of Human Skin" was retracted in 2020. Reason: duplicated images.

#### 3.2.4. The Effect of Topical SOP on the p53 Protein in the Epidermis after UVB Irradiation

The p53 protein expression in the epidermis of control group at 8, 24, 48, and 72 h was relatively weak. The p53 protein expression in the epidermis of UVB-irradiated groups at each time point was increased, and the highest p53 protein expression was achieved at 24 h. Compared with UVB group, the p53 protein expression in UVB + SOP groups at 8, 24, and 48 h was significantly decreased (*P* < 0.01), whilst there was no significant difference in the IRIDI of p53 protein at 72 h (*P* > 0.05). There was no significant difference in the IRIDI of p53 protein between UVB + vehicle and UVB groups (*P* > 0.05) (Table 1, Figure 5).

#### 3.2.5. The Effect of Topical SOP on the Epidermis Bax Proteins after UVB Irradiation

The Bax protein expression in the epidermis of control group at 8, 24, 48, and 72 h was weak. The Bax protein expression in the epidermis of all UVB-irradiated groups at all time points was increased, and the highest Bax protein expression was at 24 h. Compared with UVB group, UVB + SOP group showed significantly decreased expression of Bax protein in the epidermis at 8, 24, and 48 h (*P* < 0.05), whilst there was no significant difference in the IRIDI of Bax protein at 72 h (*P* > 0.05). There was no significant difference in the IRIDI of Bax protein between UVB + vehicle and UVB groups (*P* > 0.05) (Table 2, Figure 6).

#### 3.2.6. The Effect of Topical SOP on the Epidermis Bcl-2 Proteins after UVB Irradiation

The Bcl-2 protein expression in the epidermis of all UVB-irradiated groups at 8, 24, 48, and 72 h was significantly decreased (*P* < 0.05) compared with control group. Compared with UVB group, UVB + SOP group showed significantly increased expression of Bcl-2 protein in the epidermis at 48 and 72 h (*P* < 0.05). There was no expression of Bcl-2 protein detected in the UVB and UVB + vehicle groups at 8 and 24 h and the expression of Bcl-2 protein in UVB + SOP groups was also very weak. There was no significant difference in the Bcl-2 protein expression between UVB + vehicle and UVB groups (*P* > 0.05) (Table 3, Figure 7).

## 4. Discussion

Erythema reactions produced by skin exposure to simulated UV can be divided into immediate and delayed erythema. UVB irradiation above erythemal dose can cause skin inflammatory erythema and delayed hyperpigmentation, requiring several days to several weeks to subside. Minimal erythema dose (MED) is the amount of UV radiation that will produce minimal erythema (sunburn or redness caused by engorgement of capillaries) of an individual's skin within 24 hours following exposure. Lim et al. demonstrated that 2.5 MED of UVB irradiation increased skin EI and reached the highest value on day 2 after irradiation, whilst the skin MI was obviously increased on day 3 [14]. In accordance with this, we found that 180 mJ/cm^2^ of UVB irradiation for 3 consecutive days significantly increased skin EI on day 1 after irradiation, whilst skin MI was increased later on day 3. Topical 5.0 IU/mL and 10.0 IU/mL SOP significantly decreased skin EI in UVB-irradiated skin, indicating that a certain amount of SOP could accelerate erythema to subside. However, topical SOP of different doses made no significant difference in the skin MI of UVB-irradiated skin, indicating that topical SOP could not improve delayed hyperpigmentation induced by 180 mJ/cm^2^ of UVB irradiation for 3 consecutive days.

The article "Protective Effects of Soy Oligopeptides in Ultraviolet B-Induced Acute Photodamage of Human Skin" was retracted in 2020. Reason: duplicated images.

In this experiment, two noninvasive main indicators of skin barrier function, namely, SC hydration and TEWL, were measured. Studies found that high-dose or prolonged UV irradiation could impair skin barrier function [15, 16]. Our results showed that there was no significant change in the TEWL of irradiated groups, indicating that 180 mJ/cm^2^ of UVB irradiation for 3 consecutive days made no significant impacts on TEWL. This might be related to the UVB dose and/or irradiation method. Meanwhile, topical SOP made no significant changes in the TEWL of both irradiated and nonirradiated skin. Nevertheless, topical SOP significantly increased the SC hydration in UVB-irradiated skin treated with SOP on day 1 after UVB irradiation, however, not on days 3 and 10. Moreover, topical SOP did not increase SC hydration in nonirradiated skin. This suggests that topical SOP could not improve SC hydration and TEWL values of both normal and UVB-irradiated skin. There are many internal and external factors that could affect the SC hydration, such as water channel protein, epidermal lipids, and the quality and quantity of moisturizing factor [17]. In this experiment, topical SOP could not increase SC hydration maybe due to failure to make impacts on those possible factors.

Based on the results of our clinical study, we found that topical SOP could reduce UVB-induced erythema reaction. UV-induced erythema is related to UVB-induced DNA damage and apoptosis. When the skin receives UVB, cellular DNA directly absorbs UVB and forms light products, including a large number of CPDs [18]. Intracellular accumulation of CPDs would hinder DNA replication and transcription [19]. If CPDs cannot be repaired in time, cells with damaged DNA would be cleared through activation of p53 apoptotic pathway mechanism. In UV-induced erythema, there is infiltration of sunburn cells in the epidermis, which are apoptotic keratinocytes [1]. Therefore, we further carried out* ex vivo* experiments to explore the possible mechanisms by which topical SOP reduced UVB-induced erythema.

The article "Protective Effects of Soy Oligopeptides in Ultraviolet B-Induced Acute Photodamage of Human Skin" was retracted in 2020. Reason: duplicated images.

Acute skin photodamage caused by short-term high-dose UV irradiation can increase the amount of reactive oxygen species in the skin, resulting in DNA damage, inducing keratinocytes to undergo apoptosis and manifest themselves as sunburn cells. We detected sunburn cells using H&E and at the same time we detected apoptotic cells using TUNEL assay. We found that there were a large number of sunburn and apoptotic cells in the epidermis after UVB irradiation, which reached the highest number at 24 h and gradually reduced with time. The number of apoptotic cells detected by TUNEL assay was slightly higher than the number of sunburn cells detected by H&E staining. This might be because TUNEL assay detects the DNA breaks which occur very early in apoptosis, prior to changes in cell morphology, thus capable of detecting the apoptotic cells which cannot yet be recognized based on changes in morphology [20]. Our results demonstrate that topical SOP significantly reduced the number of sunburn and apoptotic cells in UVB-irradiated epidermis. This indicates that topical SOP accelerated removal of apoptotic cells.

CPDs are the main light product produced in UV-irradiated cells, accounting for 70–80%, and have a low rate of repair. Their absorption peak is within UVB wavelength range. Therefore, detection of UVB-induced CPDs formation and removal is important for the evaluation of DNA damage severity and repair. CPDs can occur after the skin is irradiated by UV and reached a peak after 4 h. Because CPDs removal in the skin is relatively slow, there is still a high level of CPDs in the skin 24 h after UV irradiation, even after several days [21]. In accordance with this, our experimental result showed that there were a large number of CPDs-positive cells after UVB irradiation, and the highest number was observed at 8 h, and it gradually decreased with time. Several studies found that some antioxidants, such as green tea polyphenols and retinyl esters, have a positive contribution to the removal of CPDs [22, 23]. We found that topical SOP application on UVB-irradiated skin significantly decreased the number of CPDs-positive cells compared with that of UVB group, indicating that topical SOP application accelerated the removal of CPDs. Our previous study on topical SOP effects in UVB-induced skin photodamage of mice confirmed that SOP had a strong antioxidant capacity, increased skin SOD and GSH-px activities, and accelerated removal of free radicals [10]. The positive effect of SOP may be mainly through the absorption of UV and clearance of oxygen free radicals produced from UVB irradiation, thus reducing damage caused by oxygen free radicals in CPDs nucleotide excision repair pathway. Therefore, the removal of CPDs could be accelerated through the antioxidant properties of SOP.

p53 is a tumor suppressor gene and has an important role in UVB-induced skin lesions. After p53-gene-knockout mice were irradiated by UV, the number of sunburn cells in their skin was obviously decreased compared with that of normal mice [24]. This suggests that p53 expression plays an important role in the formation of UV-induced sunburn cells. As a transcription factor, p53 protein regulates a series of downstream target gene expressions and arrests the cell cycle at G1 phase, promoting DNA repair [4]. If the DNA cannot be repaired, p53 can induce Bax activation and downregulation of Bcl-2, causing apoptosis [5, 6]. Our study showed that, after UVB irradiation, there were increased p53 and Bax protein expressions and decreased Bcl-2 protein expression compared to control group, promoting apoptosis in the dermis. In accordance with this, we found increased apoptotic cells in the epidermis after UVB irradiation. However, topical SOP application significantly decreased UVB-induced p53 and Bax protein expressions and also significantly increased Bcl-2 protein expression at 48 and 72 h after UVB irradiation.

The article "Protective Effects of Soy Oligopeptides in Ultraviolet B-Induced Acute Photodamage of Human Skin" was retracted in 2020. Reason: duplicated images.

In conclusion, our study demonstrated that topical SOP could reduce UVB-induced erythema but have no impacts on hyperpigmentation and SC hydration. Topical SOP could accelerate removal of UVB-induced CPDs and apoptotic cells through decreasing UVB-induced p53 and Bax protein expressions and increasing Bcl-2 protein expression, thereby protecting against UVB-induced photodamage.

## Figures and Tables

**Figure 1:** (a) Erythema index (EI) value in each group as detected by Mexameter MX 18 probe of MPA 9 device. (b) Melanin index (MI) value in each group as detected by Mexameter MX 18 probe of MPA 9 device. (c) Stratum corneum (SC) hydration value in each group as detected by Corneometer CM 825 probe of MPA 9 device. (d) Transepidermal water loss (TEWL) value in each group as detected by Tewameter TM 300 probe of MPA 9 device. Compared with ultraviolet B (UVB) group, the skin EI in UVB + 5.0 IU/mL soy oligopeptides (SOP) and UVB + 10.0 IU/mL SOP groups was significantly decreased (*P* < 0.05) and UVB + 2.5 IU/mL SOP group showed no significant difference (*P* > 0.05); the skin MI in UVB + SOP groups showed no significant difference (*P* > 0.05); the SC hydration on day 1 in UVB + 5.0 IU/mL SOP and UVB + 10 IU/mL SOP groups was significantly increased (*P* < 0.05), whilst that of days 3 and 10 showed no significant difference (*P* > 0.05), and the skin TEWL in UVB + SOP groups showed no significant difference (*P* > 0.05). The statistical analysis was carried out with the paired *t*-test; data were expressed as the mean ± SD for each group; ^&^ *P* < 0.001 when compared with negative control group of the same period; ^#^ *P* < 0.05 when compared with negative control group of the same period; ^*∗*^ *P* < 0.05 when compared with UVB group of the same period.

**Figure 2:** (a) Cyclobutane pyrimidine dimers- (CPDs-) positive cells in the epidermis of each group, stained by immunohistochemical staining and detected by light microscopy with ×400 magnifications. (A) Control; (B) UVB group; (C) UVB + vehicle group; (D) UVB + 5.0 IU/mL SOP group. (i) 8 h; (ii) 24 h; (iii) 48 h; (iv) 72 h. (b) The number of CPDs-positive cells in the epidermis of each group. Then, 8, 24, 48, and 72 h after ultraviolet B (UVB) irradiation, the number of CPDs-positive cells in UVB + 5.0 IU/mL SOP groups was significantly decreased compared with UVB group (*P* < 0.05); stained by immunohistochemical staining and detected by light microscopy with ×400 magnifications; ^*∗*^ *P* < 0.05 when compared with the UVB group.

**Figure 3:** (a) Sunburn cells in the epidermis of each group, stained by hematoxylin and eosin (H&E) staining and detected by light microscopy with ×400 magnifications. (A) Control; (B) UVB group; (C) UVB + vehicle group; (D) UVB + 5.0 IU/mL SOP group. (i) 8 h; (ii) 24 h; (iii) 48 h; (iv) 72 h. (b) The number of sunburn cells in the epidermis of each group. The number of sunburn cells in the epidermis of UVB + 5.0 IU/mL SOP groups at 8, 24, 48, and 72 h after UVB irradiation was significantly decreased compared with UVB group (*P* < 0.05). Stained by H&E staining and detected by light microscopy with ×400 magnifications. ^*∗*^ *P* < 0.05 when compared with the UVB group.

**Figure 4:** (a) Apoptotic cells in the epidermis of each group, stained by TUNEL staining and detected by light microscopy with ×400 magnifications. (A) Control; (B) UVB group; (C) UVB + vehicle group; (D) UVB + 5.0 IU/mL SOP group. (i) 8 h; (ii) 24 h; (iii) 48 h; (iv) 72 h. (b) The number of apoptotic cells in the epidermis of each group. Compared with UVB group, the number of apoptotic cells in UVB + 5.0 IU/mL SOP groups at 8, 24, 48, and 72 h was significantly decreased (*P* < 0.05). Stained by TUNEL staining and detected by light microscopy with ×400 magnifications. ^*∗*^ *P* < 0.05 when compared with the UVB group.

The article "Protective Effects of Soy Oligopeptides in Ultraviolet B-Induced Acute Photodamage of Human Skin" was retracted in 2020. Reason: duplicated images.

**Figure 5:** p53 protein expression in the epidermis of each group, stained by immunohistochemical staining and detected by light microscopy with ×400 magnifications. (A) Control; (B) UVB group; (C) UVB + vehicle group; (D) UVB + 5.0 IU/mL SOP group. (i) 8 h; (ii) 24 h; (iii) 48 h; (iv) 72 h.

**Figure 6:** Bax protein expression in the epidermis of each group, stained by immunohistochemical staining and detected by light microscopy with ×400 magnifications. (A) Control; (B) UVB group; (C) UVB + vehicle group; (D) UVB + 5.0 IU/mL SOP group. (i) 8 h; (ii) 24 h; (iii) 48 h; (iv) 72 h.

**Figure 7:** Bcl-2 protein expression in the epidermis of each group, stained by immunohistochemical staining and detected by light microscopy with ×400 magnifications. (A) Control; (B) UVB group; (C) UVB + vehicle group; (D) UVB + 5.0 IU/mL SOP group. (i) 8 h; (ii) 24 h; (iii) 48 h; (iv) 72 h.

**Table 1:** p53 protein expression in UVB-irradiated epidermis after topical application with SOP (IRIDI).

Group division	8 h		24 h		48 h		72 h	
	Mean score	SE	Mean score	SE	Mean score	SE	Mean score	SE
Control	0.2	0-1	0.4	0-1	0.2	0-1	0.2	0-1
UVB	2.2	2-3	4.0	3–6	2.4	2-3	1.2	0–2
UVB + vehicle	2.4	2-3	4.2	3–6	2.4	2-3	1.4	1-2
UVB + 5.0 IU/mL SOP	1.0^*∗*^	0–2	1.4^*∗*^	1-2	0.8^*∗*^	0-1	0.6	0-1

UVB: ultraviolet B; SOP: soy oligopeptides; IRIDI: immunoreactivity intensity distribution index. ^*∗*^ *P* < 0.01 when compared with UVB group of the same period.

**Table 2:** Bax protein expression in UVB-irradiated epidermis after topical application with SOP (IRIDI).

Group division	8 h		24 h		48 h		72 h	
	Mean score	SE	Mean score	SE	Mean score	SE	Mean score	SE
Control	0.4	0-1	0.2	0-1	0.2	0-1	0.2	0-1
UVB	2.8	2–4	4.4	4–6	1.8	1-2	1.2	1-2
UVB + vehicle	3.0	2–4	4.0	4–6	1.6	1-2	1.2	1-2
UVB + 5.0 IU/mL SOP	1.8^*∗*^	1-2	2.2^*∗*^	2-3	0.8^*∗*^	0-1	0.8	0-1

UVB: ultraviolet B; SOP: soy oligopeptides; IRIDI: immunoreactivity intensity distribution index. ^*∗*^ *P* < 0.05 when compared with UVB group of the same period.

**Table 3:** Bcl-2 protein expression in UVB-irradiated epidermis after topical application with SOP (IRIDI).

Group division	8 h		24 h		48 h		72 h	
	Mean score	SE	Mean score	SE	Mean score	SE	Mean score	SE
Control	2.2	1–3	2.4	2-3	2.2	1–3	2.6	2-3
UVB	0^#^	0	0^#^	0	0.2^#^	0-1	0.8^#^	0-1
UVB + vehicle	0^#^	0	0^#^	0	0.4^#^	0-1	0.8^#^	0-1
UVB + 5.0 IU/mL SOP	0.8^#^	0-1	0.2^#^	0-1	1.2^#*∗*^	1-2	1.6^#*∗*^	1-2

UVB: ultraviolet B; SOP: soy oligopeptides; IRIDI: immunoreactivity intensity distribution index. ^#^ *P* < 0.05 when compared with negative control group of the same period; ^*∗*^ *P* < 0.05 when compared with UVB group of the same period.
